# Future call for policy making to speed up interdisciplinarity between natural and social sciences and humanities in countries such as India

**DOI:** 10.1016/j.heliyon.2021.e06484

**Published:** 2021-03-17

**Authors:** Kabita Das, Biswaranjan Paital

**Affiliations:** a Post Graduate Department of Philosophy, Utkal University, Bhubaneswar, Odisha, India; b Redox Regulation Laboratory, Department of Zoology, College of Basic Science and Humanities, Odisha University of Agriculture and Technology, Bhubaneswar, India

**Keywords:** Science, Interdisciplinary research policy, Need based research, Pace in interdisciplinarity, Social science

## Abstract

**Objectives:**

Science is the erudite methodical systematic practises to study the structure and behaviour of natural objects and/or phenomena. It clearly unknot about the fact that science is a human (society) need based process that starts with social affairs, for example, need to exchange emotion and cognitive processes (psychology), feelings (literature), relation (sociology), money (economics) etc. Humanities are the use of approaches that are predominantly hypothetical but critical, and have a noteworthy historical component, and the methodical aspects distinguish it from the mainly experiential approaches of the science. The basic approaches in both remains the same that it needs a hypothesis, sound methodology, and interpretation of data. Human is the end user in both the cases. So, why only interdisciplinary research focused on the core subjects of science? For example, philosophy, deals with general and vital complications relating to matters including existence, knowledge, language, attitude, behaviour, values, ethics, reason, mind, peace and harmony in life which can be essentially a part of science (especially natural sciences and more particularly animals sciences such as zoology) or vice versa could be true. The current and future time will allow us to believe on such concept, is the main theme of the current article.

**Methods:**

Articles from all published sources are considered for answering the objective that why not concentrating to speed up interdisciplinarity. Few tables and figure are reproduced or redrawn as per the need. And numerical data are collected to present the current status of the interdisciplinarity and the need of the pace it requires.

**Results:**

It is noticed that number of research articles on interdisciplinarity in comparison to several core subject area in major databases including environmental biology are still negligible. Countries still need to inter-collaborate at interdisciplinary level for the development and benefit of human race. This needs to be done mainly at socio-economic, intercultural and scientific levels. Although numbers of steps are taken such as establishment of interdisciplinary institutes, introduction of interdisciplinary courses, interdisciplinary research and publication platforms in specialized dedicated journals, still concrete steps to introduce the course of interdisciplinarity at educational and professional level is wanting.

**Conclusion:**

Therefore, policy on pace in interdisciplinarity across science and humanities is highly wanting especially in developing countries to fix several national and international issues. Present article deals with the current status and future prospective or policies required on interdisciplinarity.

## 1 Introduction

As per the quotes of Robert James Shiller, an eminent American academician in Economics at Yale University and the fellow member at the Yale School of Management's International Center for Finance, “In the longer run and for wide-reaching issues, more creative solutions tend to come from imaginative interdisciplinary collaboration” (TRD, 2007). The story of interdisciplinarity is well approved by many stalwarts globally as it provides a platform to set novel goals and to resolve many complicated societal issues that are yet not solved by disciplinary approaches (Moreau and Mercier, 2020; Müller and Kaltenbrunner, 2019). The article is focused on the concept that why interdisciplinarity must be preferred than disciplinary approaches, for example, merging science and social science or humanities to resolve societal issues.

The etymology of the word “Science” indicates that it is originated from the “*scientia”.* The word “scienti” belongs to Latin language meaning “knowledge”. And the process of gaining knowledge deals with systematic activities used to organize information in a systematic manner about the universe. The information is gathered from a testable hypothesis, methodology, data collection, analyses, explanations and predictions about various aspects of the matters in the universe (Ajayi, 2019; Harper, 2019; Wilson, 1999, 2017; Heilbron, 2003). The above definition of knowledge leads to explain the other way meaning of the word “science”. Science is the intellectual action at practical, methodical and systematics to study the structure and behaviour to know about either physical and natural object or the world through observation and experiments. It meant to unravel the nature and its underlying fundamental mechanism(s). For example, creating different sounds (as part of language) or drawing a picture (as part of art) to exchange and understand the intention or emotion was the need of human society at prehistoric time. Similarly, starting from sending messages or video calls through different mobile phone applications, inventing genetically engineered food to rocket science, are the examples of the current day's need. Therefore, science is meant to understand the nature and fundamental mechanism of any object in the world but strictly not restricted to worldly objects, for example, studying objects out of world i.e. space science. Innovation based on need that leads to invention is the main part of science. Discovery is therefore, an essential part of it and its objective is to serve the world, not limited to mankind. It could be either the discovery of fire by prehistoric human to invention of artificial intelligence by scientist in ultra-modern era. Both the above discoveries were need based but they were made at different time points and both are applied science that belong to physical sciences. Then using fire, prehistoric man had tried to taste the test of burnt animal's body, belongs to the biological sciences. Similarly, the artificial intelligence is a combination of physical, mathematical and biological sciences (Tian et al., 2019; Uzan et al., 2019).

Science is usually grounded on methodological observations commonly called as research that is performed at different levels such as at individual, institution, government and company level. The implications of scientific research lead to change of the concept of policies related to community or society after the introduction of specific guidelines. Such guidelines usually refer to science policies. Following such policies, the output of scientific research is implemented to commercialise the products for use in daily life, in biomedical sciences, environmental protection, etc. but largely for the betterment of the earth as a single community in general and for the development of human beings in particular (Ajayi, 2019).

Currently, the human is in a stage where modern science speaks that nature is a continuum of different states of world that ranges from the physical to the chemical and finally to the biological materials and underlying principles. Current day science is formally divided into main three categories namely natural, social and the formal sciences. Natural sciences subject areas related to the core areas such as biology, chemistry, and physics. All these disciplines of science deal with nature and the natural phenomena in the broadest sense. The next branch of sciences i.e. the formal sciences usually includes subjects such as logic, mathematics, and theoretical computer science. These sciences are not based on empirical observations and for which they are sometimes are argued not to be included under science (Bishop, 1991; Bunge, 1998; Fetzer, 2013). These sciences are concept based that strengthens the natural sciences. Most of the time, the branches of natural sciences examine their concepts using logic and mathematics leading to the scope of interdisciplinary concepts. The social sciences, otherwise called humanities, deals with the study of subject areas that fall under philosophy, economics, history, psychology, civics, literature, sociology, education, etc. These branches of sciences usually aimed to deal with individuals and societies and their issues. Finally, the need based experimental oriented established results are used in society for practical use. For example, engineering, architecture, home science and medicine, are considered as applied sciences (Abraham et al., 2004; Fischer and Fabry, 2014; Engineering Technology, 2018). In fact, social branches of science usually act as the root to the natural sciences or even the formal sciences. It is because societal need acts as the mother of invention for the betterment of the human race. Many core subjects such as physics, chemistry, zoology, botany and mathematics are now becoming the sub-domain for research purposes that give the foundation of interdisciplinary science (Klein, 1990; Giles, 1992; Nissani, 1995).

The history of science goes back to the 3500 to 3000 BCE period. Data obtained from ancient Egypt and Mesopotamia in the above period gives evidence for igniting systematic scientific approaches in the human mind, although the act of hunting and invention of fire by the prehistoric people can also be considered as scientific invention (Grant, 2007; Lindberg, 2007). As per the classical antiquity Greek natural philosophy the ancient Egyptians have the major attribution to mathematics, astronomy, and medicine. A systematic attempt was noticed in them to analyse, understand, and elucidate various natural causes exist in the physical world. After the Western Roman Empire was collapsed during the first centuries (i.e. 400 to 1000 CE), various Greek philosophical concepts had lost their base in Western Europe (Lindberg, 2007). However, the recapitulation of their works was done during the rise in Islamic ages in Western Europe. These important events that lead the recovery of Greek works was believed to happen between 10^th^and 13^th^centuries that revived the ‘natural philosophy’ (Lindberg, 2007a, 2007b, 2007c). This was later on provided the base for the transformation for the scientific revolution in 16^th^ century (Principe, 2011) during which new ideas and discoveries dominated over the Greek traditional concepts on scientific facts about the physical world (Lindberg, 1990, 2007d; Del, 2016; Grant, 2007). Instrumentation and professional approaches to answer the unsolved concepts of the physical world through all the branches of sciences in 19^th^century gave a new shape to science (Cahan, 2003; Lightman, 2011). So, the previously denoted “natural philosophy” is now changed to ‘natural science’ in 21^st^ century. The “natural science” needs the help of all the branches of sciences to solve mechanisms of various concepts of the physical world (Harrison, 2015).

On the other hand, the term “humanities” is collectively used for different academic courses that usually aimed to study about the human society and culture. Nowadays, the term “humanities” is more often understood in contrast to various disciplines of natural science. Many a time it is referred as “social sciences” such as the languages (both ancient and modern), local and national literatures, political sciences, business administration, philosophy, history, geography, law, religion, culture, behaviour, psychology as well as professional training. If one sticks to the real definition of science then the above topics are nothing but an extension of human practices that co-existed from (pre-)historic time, for example, creating different sounds (as part of language) or drawing a picture (as part of art) to exchange and understand the intention or emotion. Therefore, preliminary understanding reveals that humanities are the use of approaches that are predominantly hypothetical but critical, and have a noteworthy historical component. And this methodical aspect distinguishes it primarily from the empirical data collection using systematic experiments in the (natural) sciences. However, the basic approaches in both humanities and science remain the same that it needs a hypothesis, sound methodology, analyses and interpretation of the obtained data (existing or new themes or thoughts in humanities or the obtained information form scientific experiments). Normally, the end users are the human beings in both the cases. So, why only interdisciplinary research focused on the core subjects of science? For example, philosophy, that deals in general about the fundamental analytic and predictive problems concerning matters (Das, 2013, 2016a, 2016b, 2017), can be a part of science (especially natural sciences and more particularly animals sciences such as zoology) or vice versa? Does the current time allow us to believe in such a concept?, is the central theme of this article. A clear explanation about both science and humanities provided in supplementary file may be referred for better arguments.

## 2 Interdisciplinary subjects and need based research

Interdisciplinarity is the merging of two or more than two different disciplinary concepts to achieve a common goal in research or education (Brewer and Lövgren, 1999). Therefore, interdisciplinarity which is also called as interdisciplinary studies emerged as a hot branch in both education and research (Müller and Kaltenbrunner, 2019). It is because of the successful strategic approaches that subsequently lead to achievement of the comparatively complicated goal which is usually difficult to be dealt with an un-interdisciplinary approach (Nissani, 1995). Interdisciplinarity deals with mingling of at least two or more than two academic subjects to solve a common societal issue.

For example, dealing with the length and atomic or molecular bonding pattern in a molecule, namely, deoxyribo nucleic acid (DNA), (a heritable biomolecule that governs the character of organisms), needs more physics and chemistry approaches, respectively, than biology (Ausburg, 2006). Therefore, interdisciplinary subjects such as biophysics and biochemistry have emerged to solve the molecular aspects of DNAs. A segment of DNA in the chromosome of organism's cell when it governs a particular character is called a gene. If a particular gene present in a population of a community gives rise to a particular social behaviour, for example, suicidal behaviour. Various genes such as Herpes Simplex Virus Thymidine Kinase and the Cytosine Deaminase suicidal genes (Rossignoli et al., 2019), or monoamine oxidase A gene, MAOA-L genotype (Zarogoulidis et al., 2013; McSwiggan et al., 2017; Rossignoli et al., 2019) are responsible for this unusual behaviour but it needs some social approaches first to deal the person than measuring and analysing their genetics or biochemical profile. So, for effective management in such conditions, first social approaches to identify or counsel the person is required after which biomedical or clinical approaches are required to deal with the issues with medicines and allied fields. In such conditions, interdisciplinary approaches between science and humanities subjects are more essential than collaboration among science subjects (Gunn, 1992). For example, to develop a framework for determinants of nutrition and eating in humans, it needs vast interdisciplinary approaches to find a reliable result (Stok et al., 2017).

For example, leaf-characters such as neural actions, articulating capacity, digestion, receiving neural signals, normal growth, resting behaviour, population distribution, habitat or identifying new area for migration, social cultures, social status, economic growth, personal attitude, psychological status and responses, own mental capacity control, perception capacity, though process, eating and food habits, superstitions on food habits, own physiological concepts, obesity control, hungry and hunger issues in society, time management skills, economic issues in family, society, and country, parental care, disease control, inter-cultural activities, food production and marketing, industrial revolution and inter government issues including global climate changes and other associated international issues are required to come with an idea about the determinants of nutrition and eating in human (Table 1).

**Table 1:** Main factors and examples for the development of determinants of nutrition and eating in human.

Level; stem- category	Leaf-category	Explanation	Examples of determinants
Individual; Biological	Brain Function	brain and brain functionality	dementia, orbito-frontal cortex volume
	Oral Function	oral system and oral functionality	chewing problems, wearing dentures
	Food-Related Physiology	physiological characteristics especially relevant for diet and nutrition that are not covered in the previous categories	food allergies, obesity-associated genes
	Anthropometrics	physical size and shape	BMI, birth weight
	Sensory Perception	sensory system and sensory perception	fat liking, taste preferences
	Physical Health	physical health status	medication use, chronic diseases
	Sleep Characteristics	sleep and sleeping patterns	chronotype, sleep duration
Individual; Demographic	Biological Demographics	(usually) innate demography	age, gender
	Cultural Characteristics	culturally-defined demography	nationality, ethnicity
	Situational Demographics	situationally defined demography	living arrangement, urban or rural dweller
	Personal Socio-Economic Status	socio-economic aspects of the individual	income, education
Individual; Psychological	Personality	personality traits and styles	self-esteem, personal values
	Mood And Emotions	affective states and stable moods	depressive symptomatology, positive emotions
	Self-Regulation	individual-difference traits concerned with controlling the self	impulsivity, self-control
	Health Cognitions	personal ideas and goals concerned with being healthy and eating healthily	health consciousness, healthy eating motivation
	Food Knowledge, Skills, and Abilities	personal resources relevant for diet and eating	nutrition knowledge, cooking skills
	Food Beliefs	personal thoughts and beliefs about food and eating	food ethics, trust in the food industry
	Food Habits	habits and routines around food consumption	habitual eating, willingness-to-pay
	Eating Regulation	psychological strategies for regulation of consumption	external eating, mindful eating
	Weight Control Cognitions And Behaviors	psychological aspects of weight control	body dissatisfaction, cognitive constraint
Individual; Situational	Hunger	situational occurrence of feeling hungry	hunger, food deprivation
	Related Health Behaviors	engagement in other health behaviors related to eating	alcohol consumption, television viewing
	Situational And Time Constraints	situational occurrences that impose constraints on consumption	access to a car, workload
Interpersonal; Social	Family Structure	composition and cohesion of the family/household	household size, family cohesion
	Family Food Culture Household Socio-Economic Status	food culture existing in the family/household	household food processing, family food preferences
		socio-economic aspects of the family/household	household food security, household budget constraints
	Social Influence	diet- and eating-related influences from others in the environment	peer modeling, social norms
	Social Support	diet- and eating-related support from others in the environment	social ties, community recommendations
	Parental Resources And Risk Factors	parental resources and constraints relevant for diet and eating	parental time constraints, parental nutrition knowledge
	Parental Attitudes And Beliefs	parental thoughts and beliefs about food and eating	parental food risk aversion, parental trust in food distribution
	Parental Behaviors	parental food- and eating-related behaviors	parental food habits, parental frugality
	Parental Feeding Styles	how parents go about feeding their children	parental food restriction, parental pressure to-eat
Interpersonal; Cultural	Cultural Cognitions	thoughts and beliefs related to one's cultural background	cultural values, social role of food
	Cultural Behaviors	behaviors related to one's cultural background	cultural food customs, religious rituals
Environmental; Product	Intrinsic Product Attributes	attributes intrinsic to the food product itself	product flavor, product texture
	Extrinsic Product Attributes	attributes extrinsic to the food product itself	product appearance, product price
Environmental; Micro	Portion Size	size of a food portion	portion size, visual cues to portion size
	Home Food Availability And Accessibility	availability and accessibility of food within the home	product visibility, food availability
	Eating Environment	the environment in which food is consumed	meal environment, enhanced eating environment
Environmental; Meso-Macro	Natural Conditions	natural conditions at the living location	weather, season
	Characteristics Of Living Area	the living environment	area deprivation, size of municipality
	Environment Food Availability And Accessibility	availability and accessibility in the environment	spatial distance food-consumer, neighborhood healthy food availability
	Food Outlet Density	density of food outlets in the environment	fast food outlet density, supermarket density
	Exposure To Food Promotion	presence of food promotion in the environment	exposure to food adverts, purchase prompts and food outlet
	Market Prices	cost of food	market prices, cost of a healthier basket
	Societal Initiatives	food- and eating-related social initiatives in the environment	community-supported agriculture programs, food-related NGO activity
Policy; Industry	Industry Regulations	guidelines and regulations for the food industry	nutritional composition regulations, portion-size regulations
	Industry Influence	exertion of influence by the food industry	Lobbying
Policy; Government	Governmental Regulations	food- and eating-related policies and regulations imposed by the government	food advertisement bans, subsidies for healthy food
	Campaigns	food- and eating-related governmental campaigns	educational campaigns for healthy foods, programs discouraging unhealthy eating
	Broader Governmental Policies	other relevant policies and regulations imposed by the government	immigrant-related policy, governmental health awareness

The study indicates that many factors stating form socio-cultural to behavioral and physical to physiological (all listed under leaf-category) can be influencing to alter the food, feeding behavior in human. The interesting part is multidisciplinary approaches are needed to resolve this problem rather than a nutritional approach alone (source: Stok et al., 2017).

In the study, the authors have included participants from several subjects who belong to diverse countries to reach a conclusion (Table 2). So, interdisciplinary science has not a limited scope for combination in research rather it opens a wider scope for mingling two or more subjects for a broader complexity of the society. Therefore, concepts from various social and natural disciplines may be employed to develop suitable methodology to test any societal issues that to be resolved on priority basis. It is therefore suggested to create something by thinking across boundaries, between or among various subjects based on the emerging needs of the society can be professionally managed (Policansky, 1999; José, 2015).

**Table 2:** Interdisciplinary participants to across various countries to evaluate determinants of nutrition and eating framework.

	Workgroup members *(N=87)*	External experts *(N =* 129)
Division of age group expertise	• 15% children • 65% adults • 20% elderly	• 30% children • 57% adults • 13% elderly
Scientific backgrounds	• Anthropology • Biology/Human Biology • Dietetics • Economics • Epidemiology • Food Engineering • Food Science • Food Technology • Geriatrics • Health Promotion • Marketing and Consumer Research • Medicine • Nutrition Science • Pediatrics • Physical Education • Physiology • Physiotherapy • Psychiatry • Psychology • Public Health • Social Demography • Sports Sciences • Statistics	• Biology/Human Biology • Biometry • Economics/Health Economics • Educational Sciences • Environmental Science • Epidemiology • Food and Nutrition Science • Genomics • Geography • Human Ecology • Human-Computer Interaction • Marketing • Mathematics • Medicine • Nursing Science • Policy • Psychiatry • Psychology • Public Health • Sociology • Sports and Physical Activity Science • Statistics
Countries	• Belgium • Finland • France • Germany • Ireland • Italy • Netherlands • Norway • Poland • Spain • United Kingdom	• Germany • Italy • Belgium • Netherlands • France • Ireland • Finland • UK • Denmark • Austria • Poland • Switzerland • Marocco • United States

The table describes about the framework required for the heterogeneous participants (interdisciplinary background) to develop determinants of nutrition and eating. The authors have opined that without the interdisciplinary onion it would not be possible to make a framework for determinants of nutrition and eating. (Source: Stok et al., 2017).

Outsized engineering teams are typically interdisciplinary in nature, as a part of them it needs to handle power stations, some need to handle infrastructure, some need to handle security etc. So, bigger projects usually require the melding of several specialties. A beautiful example can be given when an operation is made in a hospital. A team of different clinical specialists such as anaesthesiologist, neurologist, surgery experts, haematologists and the concerned organ specialist are required to have a successful operation. To build a home, specialists such as astrologer for orientation of the home architecture, an engineer to sketch the design and to build the house, carpenter, painter, electrical expert etc are required. Without a single expert, a beautiful home can't be made or completed. So, “interdisciplinarity” is a need based approach from education and research to practical utility in society. However, the term "interdisciplinary" is found to be many a time narrowly used in academic sectors, while its broad meaning tend to use it in many sectors starting from surgery in hospitals to environmental management (Shrestha and Bhadra, 2019; Voarino et al., 2019; Bruzzese et al., 2020; Khoza-Shangase et al., 2020; King et al., 2020; McHenry et al., 2020; McKee et al., 2020; Moreau and Mercier, 2020). However its confined use in educational sectors is basically limited to training pedagogies in teaching learning systems. It is primarily based on the use of the concepts of various accepted modern or conventional subjects in academics (Edge et al., 2013).

The processes of interdisciplinarity constitute the learners (can be students or teachers or community in society), researchers (concentrating the contemporary problems of society at language, communication, health, medicine, education, care and all other aspects of human life. Objectives pertaining to environment, wild and human life need integration of professional and technological inventions to fulfil a common but difficult goal (with disciplinary approaches) can be resolved easily with interdisciplinary approaches (Ali, 2011). For example, the complex problems such as origin of epidemics or pandemics such as SARS or mers or HIV, or climate change issues such as rise in CO_2_ level, temperature, glacier melting needs various interdisciplinary as approaches from clinical, pharmaceutical, environmental, social and computational and physical sciences to be solved. The current case of the COVID-19 pandemic is the bright example where clinical, environmental and social approaches are suggested (Das et al., 2021a; 2021b; 2021c; Das and Paital 2020a; Mousazadeh et al., 2021; Paital, 2020; Paital et al., 2020a; 2020b; Paital and Agrawal, 2020). One needs to identify the issues with temperature rise, meanwhile, another need to address the frequency of the occurrence of the disease and its mode and speed of transmission. Sometimes such a strategy becomes a miracle to strengthen a dying subject or neglected unsolved issue (Oakland University, 2019). Interdisciplinarity is strongly suggested to be employed where the field or matter is already fingered to be neglected, misunderstood or misinterpreted and avoided due to its unachievable nature by conventional disciplinary approaches, for example, rural literacy, women education and tribal ethnic studies or even some core social science subjects such as philosophy and history in many Indian Universities (Das and Paital, 2020b).

On the other hand, interdisciplinarity can also be similarly applied to understand the underlying complex mechanisms of few disciplines possible by merging their concept and perceptions (Lindvig and Hillersdal, 2019). The term interdisciplinary as adjective is mainly confined to educational hubs to make the teaching learning system easy especially to make the pupils to understand the universal but subject specific events though muti-aided (from various subject specialities) pedagogy programs (University of Texas, 2017; Mäkinen et al., 2019). For example, an on touched area of research in India is correlating between the haematology (blood cell pattern) and proteomics (study of proteins present in a particular community) of women from a particular race or community with any malfunctioned social activities such as their strong attitude to collect dowry during marriage and to torture newly married girls. Therefore, the gradual need of the comprehensiveness of interdisciplinarity is believed to be made spanning the social sciences, natural sciences, humanities, and professions in interdisciplinary research, education, and health care (Klein, 1990).

Although the term “interdisciplinarity” is recurrently used as the most eye-catching word in various fields in 21^st^ century, the perception about it has antique backgrounds, mostly goes back to Greek Philosophy period (Clark, 1999; Frodeman, 2010). JT Klein (1990), one of the international experts on interdisciplinary studies from Wayne State University states that “*the roots of the concepts lie in a number of ideas that resonate through modern discourse-the ideas of a unified science, general knowledge, synthesis and the integration of knowledge*”. Similarly Giles (1992) opines that “*Greek historians and dramatists detects that mechanisms from other realms of knowledge from unrelated subjects such as medicine or philosophy can be considered to further understand a materialistic phenomenon*”. In general, it indicates that both clinical science and humanities need to be merged together to study the materialistic world, not with any of the above alone. Therefore, a general opinion comes as “*any broadminded humanist project involves interdisciplinarity, and history shows a crowd of cases*” (Gile, 1992) and one of the paramount example of such theory was deduced by Leibniz's in 17^th^ century and as per his opinion “*for a system of universal justice, inputs from linguistics, economics, management, ethics, law philosophy, politics, and even sinology are required, putting a stepping stone for interdisciplinarity across the boundaries*” (Smith, 2004; Frodeman, 2010; Newlands, 2010).

As per the oxford dictionary research is defined as “the systematic investigation into and study of materials and sources in order to establish facts and reach new conclusions”. Therefore, accepting “*everything is* granted” is essentially considered as an excluded part of research; rather, the fact needs to be believed based on observations”. Nowadays, the addition in the definition is made that any research needs to be need based. For example in market research, if it has long been recognised that a product costs less to retain existing customers than to attract new ones, one has to ensure that what is important to the customer before the customer's, are fulfilled with the new product or not. To know it, data systematically need to be collected from the market to ensure that data is actionable. In such conditions, understanding about the features of the products, need of the tangible and intangible aspects of customers, customer satisfaction, and product price is needed to identify gaps for increasing product quality. And also it gives an idea of the performance of the current product as well. After ensuring everything, the investment may be made so that improvements will have the biggest impact.

Citation of above example indicates that in commerce or similar products in all disciplines of science and humanities starting from home appliances to books and intellectual products follow a similar pathway. Therefore, a need-based analysis about the custer and the product is equally important to prioritize feature development and investment. Such analysis indicates, “generating new products is required which must be need based”. For such research, an interdisciplinary approach gives a huge clue for the analysis. For example, current day societal needs, identifying good products as per need based using statistics, is the need based research. Therefore, recent studies indicate that interdisciplinary research has its own benefits to the society over any disciplinary researches (Shrestha and Bhadra, 2019; Voarino et al., 2019; Bruzzese et al., 2020; Khoza-Shangase et al., 2020; King et al., 2020; McHenry et al., 2020; McKee et al., 2020; Moreau and Mercier, 2020).

## 3 Present day need: the interdisciplinary research

Of late there is a buzz on the term “interdisciplinary sciences”. Few scholars argue that it is not a new branch but is a repeatation of the old fashion in science that was done till 19^th^ century. It is a completely new emerging branch in various fields of sciences and humanities that needs to combine. It is advocated that such a combination can better exploit the social issues toward a grand solution. There is nevertheless another advantage that exists in humanities. Yet, unlike the sciences, humanities have no central discipline. This makes it easy to merge any humanities discipline with any science discipline to form a new emerging hybrid discipline. Various examples are given in the previous section to explain the advantages of interdisciplinarity. Therefore, it raises a simple question. At the present day, that do one needs to introduce such interdisciplinary subjects at school or college even at university level; education in developing countries such as in India or even in developed countries such as the USA or UK?

In response to the above questions, it was again questioned to teach science in schools and colleges as different subjects such as physics, chemistry, biology and mathematics. That the course must be designed to teach the biology of evolution and nutritional value of an apple, and finally, how apples ripe following hormonal and biochemical changes but finally follows Newtonian mechanics while they fall from the tree. It is not confusing; rather statement meaning how Newtonian motion is an applicable movement of molecules inside a cell, thus indicating a biological application of physics, must be taught to the students. On the other hand, how evolution of biological molecules in earth (for example cosmic theory of evolution for the creation of earth for the creation of nucleic acids, nucleoproteins etc) makes them adapted to discharge a particular role be explained to students, implicating physical function in terms of biology. Such concepts make them able to understand that Newtonian mechanisms can even applied inside the cell to various cellular events such as cell cyclosis or cytoplasmic streaming. Using Carbon dating (belongs to partly chemistry and physics) is also used to understand the biology of evolution. Calculus, determinant, integration and matrix are used to study numerical genetics promptly. When the working community including researchers and students will be able to understand the need for such approaches, interdisciplinarity will stand alone globally. In India, the concept of biology very rarely utilises the concepts of physics and mathematics but when combined, resulted into a powerful and useable tool as per the need of the society (Ali, 2011).

It is not very difficult to have an association among disciplines of science and humanities. The effort although not reached up to expectation, seems to have started long ago. For example, BAG Fuller, a philosopher, has discussed very nicely about the very fundamental concept of atoms (chemistry and physics). He describes the “*elements reduced to atoms*” as per the Leucippus and Democritus pulverised “*what really is into an infinite number of atoms Eleatic (relating to Elea, an ancient Greek city in south-western Italy, or the school of philosophers that flourished there in about the 5*^*th*^ *century BC, including Xenophanes, Parmenides, and Zeno) in their internal character and devoid of all qualities and differences except those of size and shape. All the atoms are everlastingly in motion of their own nature flying about here and there and it is due to their clustering and dispersions and to the formation of vertices by the component motion of their collisions that universes are generated. This generation is entirely “mechanical” and un-purposive, controlled and directed only by impact with resultant agglomeration and modification of movement unlike Empedocles, Anaxagoras, Leucippus and Democritus considered change of place in a plenum impossible, and asserted the equal reality of the void or the empty space*” (Fuller, 1969). Possibility of understanding the atomic phenomena in an element although not fully understood but very nicely represented by a philosopher about five decades ago when electronic revolution for social interaction even had not touched its initial target.

Now with easy access to every form of knowledge via electronic media, interdisciplinarity is quite certainly achievable (Rutherford et al., 2009; Clark and Wallace, 2015). Access to computer or internet forces many to remember facts in brain. Although soft copy storage devices make them less curious to remember huge information, it opens an easy path for interdisciplinarity with all information in one hand. In such cases a deep knowledge on a specific discipline is suggested that really questions about interdisciplinary science. However, it is quite easy at this time point through introducing interdisciplinary subjects at school and college level studies. As a key resource, information (memorised raw concept) in the form of knowledge (practised method) that is required economic and social progress will lead to a knowledge based society. Curiosity in understanding and management of “interdisciplinary knowledge” via education and professional training although increased lately but now seems achievable. The reason for the late pickup for an interdisciplinary knowledge society, or the informational society, could be due to its complexity, integrativity, reflexivity and interpretation. However, through both the formal, non-formal or informal education building a pillar for interdisciplinarity is possible.

Interdisciplinarity gives a new approach to the world. The changes at socio-cultural level, scientific developments and socio-political and socio-economic level can only be understood with interdisciplinary mode. An education or training based interdisciplinarity through science and technology by promoting partnership with humanities is essential. It must have an objective to accept the advancement and superiority from that of the conventional mode of disciplinary approaches in the current day society regardless of the pure disciplinary conceptualisation. In cases, the differences in social race, ethnic group, religion or nationality may put interdisciplinarity on back log to achieve the common goals, for example, solving the problems of food security in all developing and under developed countries. The implementation of new technologies based on interdisciplinarity, needs continuous and extensive effort equally by the organization, teachers and students and finally, nearby society. So, both classroom and society are the best platforms to start and implement interdisciplinarity, respectively. Since interdisciplinarity is the needs of our society, new technologies and curriculum based teaching learning offers students to learn at their own pace about it. It will enable them to use newer knowledge in interdisciplinary mode to solve the complex problems with more efficiency and also to transfer the same knowledge to others. Interdisciplinary knowledge must be used at personal, community, society and county or international level, therefore not only to deal to collect, uses and transfer the knowledge but also to preserve the knowledge safely. As usually, the teachers have the key role to play, therefore, they must undertake the major responsibility in the journey. It is because the attitude of a teacher towards using new tools, technologies and methods of teaching and transforming a disciplinary classroom to interdisciplinary classroom will decide its path. So, merely, implementing and incorporating interdisciplinarity in the educational process may not solve the issue to achieve the goal (Vali, 2013). The programs for continuous interdisciplinary professional training that must be useful to both students and teachers involved into the educational play (through interdisciplinarity) in the platform (society) is needed. Since a country's future is usually decided in the classroom, interdisciplinarity will be easy to achieve by introducing the courses from schooling time.

Even though interdisciplinarity appears to have various difficulties at the ground level, multiple solutions may also be derived to resolve the key problems to interdisciplinary studies. As one of the key solutions, all school pupils can be educated in science under a single discipline. With such an approach, students can be trained with every elementary topic of physics along with a concept of how under specific circumstances physical objects interact with or among each other to end up with different products. While drawing such concepts, automatically the new products will deal with the concepts of chemistry. And gradually, the students can be discussed to learn how various elementary chemicals such as carbon, hydrogen and oxygen interact with each other to form complex organic molecules. At such juncture of teaching, a turn towards interactions among organic chemical compounds such as enzymes, proteins, peptides, nucleic acids, glucose, fructose and sucrose and large and small lipids were interacted and self-organized to form the biological system which is nothing but an extension of physics and chemistry.

Further at the college level, students have to be taught science with additional wisdom on it so that they may penetrate into specific disciplines of their choice but with elementary knowledge on each discipline. The whole strategy shall be to execute how pupils will acquire knowledge on various key rules and concepts of physics, chemistry, botany, zoology, mathematics under single subject avenue. Eventually, at the hierarchy in the teaching learning system, pupils need to acquire enough depth in a particular discipline or sub-fields of any discipline with a background of interdisciplinarity for the purposes of research at postgraduate level (Frodeman, 2010). Such plans need to be done to merge humanities with science subjects as well. Following such emerging policy, pupils will be able to expand their vision and understanding to move with research activities in higher hierarchy of educational niche with interdisciplinary or transdisciplinary approaches. They will understand the language of all disciplines and with such knowledge, collaborations for interdisciplinarity or transdisciplinarity would be more efficient. With such a stepping stone towards interdisciplinarity, collaborations amongst researchers with comprehensive familiarity on science as a whole or in combination with humanities would help for pushing research on the frontier issues of society in all possible aspects. As a result, it may lead to resolve the complicated issues of society with multi or trans-disciplinary approaches rather than disciplinary approaches (José, 2015, Figure 1).

**Figure 1:** Representing figure showing the need of improving thought process for interdisciplinary approaches rather than on a single thought process to solve the problems of the society (adapted from The Open University, American Psychological Association, Kendall/Hunt Higher Education, zozoovodafone, India, all images were downloaded from Google images with above citations are acknowledged).

## 4 Recent advances and lacuna in interdisciplinary research

### 4.1 Articles published on interdisciplinarity

As per Machiel Keestra, the main problem rests under the strong disciplinary mind-set of many by using existing or stimulated generative technologies and it mainly aimed to solve recent complex societal problems. Mainly four things would act as the key drivers for the interdisciplinarity, 1. Disciplinary structure of the university, 2. Disciplinary structure of academic education, 3. Organization and funding of research and 4. Publication culture and peer review process (Keestra, 2013). Owing to the above objectives on the importance of interdisciplinarity, it has been noticed that a growing interest has been paid to it. A search on the term “interdisciplinarity” in PubMed, one of the largest databases of the world scholarly articles, indicates that a gradual increasing attention of researchers was paid on it from 1950 until now. Revolution of instrumentation and different concepts such as unravelling DNA molecules and central dogma of body physiology i.e. DNA-RNA and protein synthesis after the 1950s could be the reason attributed behind it. The number of articles on “interdisciplinary” has picked up pace after the 1980s, being the highest number of articles published in PubMed was in the recent decade i.e. from 2011 to 2019 (Figure 2a). Only, 1, 2, and 6% of the total articles on interdisciplinarity was published in the years 1971-80, 1981-90 and in 1991-200, respectively, whereas, 91% of the articles on interdisciplinarity were published in the recent decade, indicating its importance in the current day society (Figure 2b).

**Figure 2:** Articles published on interdisciplinary in PubMed. a. Number of articles published in PubMed on “interdisciplinary” from the year 1990–2019. b. Percentage of the article published PubMed on “interdisciplinary” from the year 1990–2019 (data source PubMed, accessed as on 11.08.2019 supplementary figure 1).

Interesting featured articles published in “Nature” indicates that from mid-1980s, people have increasingly started to cite papers that come out of their own disciplines (Van Noorden, 2015a, 2015b). The author tried to use the name of the journals from 35 million papers from Web of Science to create 14 major conventional disciplines (such as biology or physics) and 143 specialities. Results of the authors’ study indicate that the portion of article references that aimed to identify researches done on other disciplines is elevated in both the natural and the social science subjects. In contrast, the portion that aimed to point any sub-discipline in the same speciality, for example, a genetics paper pointing to zoology or botany, work on events on ancient society pointing to history etc gained an alleviating trend. On one hand, although a major concern was raised that a little interdisciplinarity is better to start than a too much interdisciplinarity to be picked up at a time, so that articles that combine very distantly related fields may lose the chance of high citation.

On the other hand, irrespective of citations of articles, intensive interdisciplinary works have better and broad societal and economic impacts in society than disciplinary works (Noorden, 2015a, 2015b). It is because; the results obtained from interdisciplinary approaches are solid and their impacts are much stronger than disciplinary results. One compulsory need for interdisciplinarity to be successful longer time is usually required to understand and implement interdisciplinary results in society in the form of policy/tools/technology. From, 1910 to 1950, it was noticed that social science and humanities ranked over engineering and natural science in terms of citation with the term “interdisciplinary” in their title which was then declined in favour of the former categories. Exactly, humanities and social sciences have scored within 0.01% citation whereas the former category ranged approximately from 0.07 to 0.05 % citation, out of all articles published during the above specific period. India has topped the list in publishing the interdisciplinary articles where as Germany lagged behind in the list (Table 3). It is clear from Table 3 that most of the developing countries give importance on interdisciplinarity to grow faster or to clean their societal issues. On the other hand, the change in average citation of the articles with respect to time scale was less in humanities articles in comparison to the pure science articles (Noorden, 2015a, 2015b). However such analyses are lacking on the interdisciplinarity between any hybrid subjects between science and humanities.

**Table 3:** Country wise interdisciplinarity research publications out of total articles published.

Serial number	Country	% of interdisciplinary articles published
1	India	13.00
2	Main Land China	12.40
3	Taiwan	11.90
4	South Korea	11.20
5	Brazil	11.00
6	Italy	10.30
7	United states	9.700
8	Japan	9.700
9	United Kingdom	9.10
10	Germany	8.50

### 4.2 Recent researches on interdisciplinarity

Interdisciplinary research, publications and their citations are quite different from any disciplinary work (Yegros-Yegros et al., 2015). The authors have considered few of the published papers in various journals and reached the above conclusion (Table 4). Contributing to the importance of interdisciplinarity, many recent works have attributed to different aspects of societal issues mainly to the health care system. Joachim et al. (2019) opined that the health workers especially the young doctors are not convinced with the disciplinary training they have obtained to practice in hospitals. For example, one need a training from physics to handle ultra sound or x-ray machine or to operate using modern equipments. On the other hand, in practical cases, many clinical issues need interdisciplinary approaches. In healthcare systems, especially in women during pregnancy, a team work among psychologists, haematologists, gynaecologists with anaesthetic and obstetrical teams is needed in an excellent interdisciplinary mode of action (Pytel et al., 2019). In such conditions an interdisciplinary multimodal pain therapy is suggested to be delivered in a personalized, mechanism- and goal-oriented manner on the basis of an individual case conception (Grolimund et al., 2019). Before a personal or community based health care intervention, interdisciplinary approaches to study the psychology of patients is highly suggested (Wendt et al., 2019). Early assessment of health of a community by a multidisciplinary team to avoid any emergency in health care intervention is required (Cassarino et al., 2019). Then only large social development with interdisciplinarity will be achieved (Lindmark et al., 2018).

**Table 4:** Effects of citation in interdisciplinary works (Source: Yegros-Yegros et al., 2015 under creative common attribution license).

	Steele & Stier (2000)	Rinia et al. (2001)	Adams et al. (2007)	Levitt & The!wall (2008)	Lariviere & Gingras (2010)	Uzzi & al. (2013)	Lariviere & al. (2015)
Sample	750 articles in	All academic	Articles from two	All science and	All papers	All papers in	All papers in WoS
	forestry (1985-	groups in physics	UK universities	social science	published in	WoS (1990-	(2000–2012)
	1994)	the Netherlands		articles	WoS in 2000	2000)	
Database	*Journal Forest*	WoS	WoS	WoS and	WoS	WoS	WoS
	*Science*			Scopus			
Unit of analysis	Article	Journal	Article	Journal	Article	Article	Co-citation
IDR Indicator	Brillouin's	% papers not	Shannon diversity	Number of	% cited refs. to	Median	Dichotomous:
	diversity index	published in	& % cited refs. to	disciplines	other SC	disparity, 10%	Intra. vs. Inter
		physics	other SC	assigned to journals		percentile disparity	subsdiscipline
Aspect of diversity	Combination of variety and balance	Balance	Combination of variety and balance	Variety	Balance	Disparity	Disparity
Measure of	Average annual	Normalized	Normalized	Normalized	Normalized	Not normalized	Normalised
citation impact	citation rate	indicators	indicators	indicators	indicators		indicators
Correlation	Positive	No effect	Visual evidence	Negative effect	Inverted U	Low median	Mainly positive
IDR vs Impact			of inverted U	in some disciplines	shape	disparity, with high 10% disparity	
Regression controls	Yes	No	No	No	No	Yes	No

Similarly in health sciences, a solid personalized planning with interdisciplinary multimodal pain management is suggested in patients. Psychology of the patients is important to understand for a multidisciplinary pain management to be done in such cases (Grolimund et al., 2019). Many indigenous communities are found with the superstitious philosophy with traditional substances that they use for the treatment or for the prevention of diseases. Although advanced, effective and viable solutions are available to them as alternative and promising sources for prevention and treatment. Yet such traditional communities are concerned about their superstitious thoughts for the treatment of mental and physical health. Such communities are the best sectors to employ interdisciplinarity. Whole community outreach program with multiple experts are needed to carry out research and finally, coordinating, monitoring, evaluation and follow-up of such research needs a highly interdisciplinary program. Such research should be pertaining to substance use problems that need to be conducted with and by indigenous communities for better health care (Wendt et al., 2019).

An interdisciplinary research agenda is also proposed to study and design preventing measures for suicide in different communities across the world. Such approaches are more based on social sciences (counselling), also dependent on physics to design the ceiling fan in such a way to make the attempter fail to suicide the fan will be over loaded to be collapsed (Kariippanon et al., 2019). The latter needs the use of the concept of physics along with little biology. Similarly, an interdisciplinary approach is suggested to prevent the negative influence of co-morbidities on the quality of life of multiple sclerosis patients. Such cases are evident across the world (Goischke, 2019). In cancer patients, drug-dose, mental care, pain care, social acceptance, medication access etc. are highly essential. So, holistic research approaches are needed to progress the easy life in cancer patients (The Cancer Research UK, 2019). In medical discipline itself, an urgent interdisciplinary approach is needed under emergency conditions such as under cardiac arrest or coronary artery disease associated with other issues (Busch et al., 2019). Dedicated professional with social and medical background with proper counselling knowledge is needed to give the patients early treatment in complications observed beyond the level of clinical approaches, suggesting recruitment of interdisciplinary social and health care personals in hospitals (Cassarino et al., 2019).

Breakthroughs in research are considered problems of the society are analysed from all angles and solved from a new perspective. This is possible when an outsider thinks of the problem from its own insight. It gives a stepping stone to interdisciplinarity. Indeed, all disciplinary researches are frequently relying on experts from their own fields but really need expertise from different disciplines. For example, projects in biological sciences such as genetics, biochemistry, molecular biology, protein chemistry, or metabolomics increasingly rely on biologists but at the same time working with experts in data mining and machine learning is also needed, for example, to use advanced techniques such as mass-spectrometry, databases in such area. Therefore, developmental biologists, medical researchers, chemists and physical science workers need to work together with mathematicians to invent new algorithms in synthetic biology to interface the above subjects to make lively processes easy. For example, people from medicine, teams of chemists, biologists, and clinicians may design specific nanoparticles to counter a particular deadly preirn for the treatment of cancer. When such collaboration is accomplished among multidisciplinary teams effectively working together, the result is used for massive benefits for society (Hall et al., 2008; Owen et al., 2012). So, interdisciplinary communication skills are becoming an emerging and core area for both social and natural scientists. Landing on mars, moon, sequencing the whole human genome, and the discovery of nano science can be merged for the betterment of the society (Dahm et al., 2019). So, a transition of knowledge from discipline to interdisciplinary seems to be the present day of the society starting from health care to social services (Lindmark et al., 2018). However, still merging humanities with science is a paradigm in the present society.

### 4.3 Interdisciplinary journals

As per Machiel Keestra the fourth key drivers for interdisciplinarity is publication culture and peer review process of interdisciplinary studies (Keestra, 2013). Experiencing such lacuna, many international publishers came forward with specialised journals to support such studies. For example, Measurement: Interdisciplinary Research and Perspectives, started in 2003 by Taylor and Francis, “Minerva”, “Policy Sciences” and “Scientific Reports” a multidisciplinary journal published by springer Nature group and also its Journal “Nature” has asked for a special issue on interdisciplinarity (Anonymous, 2015).“Social Welfare: Interdisciplinary Approach”, the prestigious journal “Science” published by American Association Advancement for Science, “Current Science” published by The Indian Academy of Sciences, “PLoS One from Public Library of Science, USA etc. are few to name them. Most surprisingly many journals also publish from the subject areas from both humanities and sciences, giving a positive clue for the advancement of interdisciplinarity that will fulfil the real need of the society. Heliyon, the recently published journal by Cell Press (Elsevier) provides ample scope to publish highly specialised motivated articles on interdisciplinarity mode.

### 4.4 Role of universities and organisations

To bring interdisciplinarity up to level, many universities and organisations across the globe have opened new department's to teach interdisciplinarity. For example, University of Southampton, UK for creating synergies, tackling global challenges, has opened Interdisciplinary University Strategic Research Groups, OakLand University, Rochester, USA fixed its mission for interdisciplinarity and formulated “The Association for Interdisciplinary Studies (formerly Association for Integrative Studies), an interdisciplinary professional organization founded in 1979, “Banaras Hindu University, India and Indian association for The Cultivation of Science, India have also their Interdisciplinary centres, Cambridge University, UK, has also interdisciplinary centres in the subject areas of cancer, conservation, energy, global food security, language science, etc,. In a recent event, to bring research in social sciences with the help of science subjects, the University Grants Commission (UGC), the largest university funding agency of India, has recommended creation of a Humanities research board termed as “Social Science/Humanities Research Board” after setting the “Science and Engineering Research Board” with special funding for research in social and allied sciences (Balaram, 2019). “The Board may introduce special initiatives which promote inter-university collaborations along the lines of existing inter-university centres set up in specialised areas of science,” UGC added. UGC has also approved new need based applied courses such as Things (IoT), Artificial Intelligence (AI), Robotics and many more. For a University in Agra, the UGC has approved Bachelor in Vocational (B. Voc.) Degree for AI, Robotics and IoT. In another university, in Coimbatore, the Commission has approved B. Voc degree program in AI and Machine Learning. In JAIN (Deemed to be University), in Bengaluru, the Commission has approved certificate courses like Digital Marketing Fundamentals, Fundamentals of Patents, Private Banking and Export and Import Documentation (Bangalore Mirror Bureau, 2019), adding another feather for modern sciences but with interdisciplinarity. However, a hybrid subject by merging pure science with humanities is still missing.

Adding one feather to the idea of interdisciplinarity, University Grants Commission, the leading governing body for the under graduate, post graduate and Philosophy in Doctorate courses in India, has implemented the choice based credit system (CBCS) at college (bachelor level studies) level. It is a widely adapted (for example, 5666 private and government colleges of the state Odisha, follows this system) and wonderfully designed syllabus that allows the students to opt any of the interdisciplinary subjects under elective course along with a core subject. For example, a student having physics as a core subject can opt history, philosophy or economics as elective subjects in a three years undergraduate course. It must be helpful to pupils to have a wider knowledge on interdisciplinarity rather only expertise on their core honours subject is the central idea behind introducing CBCS system (CBCS Syllabus, 2019a; b).

## 5 Gaps and policies needed for pace in interdisciplinarity

In the 1920's, technological and social scientific demands prevailed in society for interdisciplinarity. Using the Social Science Research Council (established in 1923 at New York, USA) as a stem, such changes were deliberated after World War II. However, the problems seemed to be persisted and achievable steps were lacking in interdisciplinarity. The Organisation for Economic Co-operation and Development (Paris, France) reported in 1972 that in interdisciplinarity, problems of teaching and research in Universities are a large concerning factor. Association for Interdisciplinary Studies, (formerly known as Association for Integrative Studies), was established to short out the gaps present in interdisciplinary studies. It was an interdisciplinary professional organization founded in 1979 to promote the interchange of ideas among scholars and administrators in the disciplines of and sciences humanities. It has started working efficiently on the issues, indicating lack of expected advancement in interdisciplinarity. And adding to the concept that “still educational system lack in interdisciplinarity and further steps are needed”, International Network for Interdisciplinarity & Transdisciplinarity was established 2011 in collaboration among US-based Association for Integrative Studies, the European-based Transdisciplinarity-Net, and the Center for the Study of Interdisciplinarity at the University of North Texas in the US (Keestra, 2013). A meeting was held in New York City among the above to form network and the mission was by the International Network for Interdisciplinarity & Transdisciplinarity (INIT). It was launched after observing the fact that the subjects of interdisciplinarity and transdisciplinarity are quite diversified and they consist of various subgroups. Most importantly, each subgroup is with its different strengths, emphases, applications, and perspectives but could be merged to achieve a common goal. As per INIT, it would ease communication and collaborative work among organizations, institutions, communities and individuals with a view of inter- and transdisciplinarity as a vibrant way to respond to the challenges of 21^st^ century society. Seminars, workshops, and conferences will be held to inaugurate this community and to develop a common agenda” (INIT, 2012).

Many organisations and Universities later on have opened special departments on interdisciplinary studies and tried to associate multiple disciplines across the subject boundaries. It was observed that although interdisciplinarity has limitless boundaries to resolve the most complicated issues of the society, researches using interdisciplinary approaches have not reached up to expectation. It is because, the terms such as “science”, “humanities”, “science and humanities”, “interdisciplinary” and “interdisciplinary research” are queried in major databases including Google, Google scholar and PubMed, the result was discouraging. Number of articles or hits found to have a negative trend line with a high degree of decline in the order of the above term mentioned (Figure 3). For example, the trend for the number of hits (that may broadly indicate the works or articles present in respective databases) with the above terms in the order they are mentioned had negative correlation coefficient values such as -0.86 (Figure 3a), -0.83 (Figure 3b) and -0.71 (Figure 3c) for PubMed, Google Scholar and Google, respectively. Since above integers are approaching the highest correlation coefficient values i.e. -0.9, the difference among the number of hits or the trend line observed are with high statistical significance. It clearly indicates, still interdisciplinary research has to march a lot to establish its ground. Especially, in developing countries such as India although excels well in terms of interdisciplinary publications, such collaborations are highly wanted. Researchers across the disciplines such as from science and humanities therefore should come forward to join hands for multi- or transdisciplinary approaches. Funding agencies also need to pay attention to ask for such projects from the researchers on priority basis.

**Figure 3:** Number of articles or hits obtained in Public Library of Medicine (PubMed), Google and Google scholar using key words science, humanities, science and humanities, interdisciplinary and interdisciplinary research. a. Number of articlea (hits) in Google, b. Number of articles (hits) in Google scholar and c. Number of articles (hits) in PubMed.

Due to multi-approach problem solving systems, interdisciplinarity is now the focus of attention for many institutions that promots teaching learning, skills, organisational and social entities concerned with higher education. As per the Ali (2011), although interdisciplinarity has been paid the most attention nowadays for which it is named “interdisciplinary higher education” practically, it is facing multifaceted criticisms, obstacles and challenges. Mainly, the challenges are with subjects in humanities for example in language and philosophy subjects, because they lack evidence based data, (mathematical/statistical) analyses, interpretation and conclusion. The difficulties faced are mainly at cultural, organisational and professional level (McEvoy, 1972).

A self-studied (by the authors) unpublished data in different Indian Institutions across the country reveals that at professional level, the first limitation in interdisciplinarity is the training of the researchers strictly on traditional disciplines. This limitation in interdisciplinary ventures makes it impracticable to sole disciplinary knowledge. For example, a discipline that has specificity for more quantitative "thoroughness" may yield a practitioner who has a belief that they and their discipline are comparatively "more scientific" in comparison to other disciplines. Undoubtedly, the scientific experiments and their outputs are universally and highly essential in life. At the same time, numerical data from science subjects cannot resolve the issues of the society that are associated with values, love and emotion in life. And, without ethics, values, love and emotion, life is ineffective and, is well addressed by humanity subjects. Therefore, such concepts have to be understood by the researchers from both disciplines and there is no harm working together. Physics and philosophy are considered to be two examples for the former and later cases, respectively (Das and Paital, 2020b). In such cases, the problem solving skills of the researchers from the former discipline always depend on quantitative approaches. Under this condition, a pin pointed portion of the problem is cleanly solved or answered. As a result, such approaches lack to solve a problem from broader dimensions. For example, analysing and determining low income as the factor for yielding a mentality of people demanding dowry from the daughter-in-law side or vice versa loses its chance to unravel other socio-economic factors. Some of the factors listed are, strong inclination towards old customs (mandatory to collect dowry), social pressure (society draws a bad impression if dowry is not collected or given), prestige issues (if dowry not given, people remarks them as low cadre community), and cultural (if dowry is not given/collected, an ancient cultural system will be lost, god will get angry, cultivation yield will be restricted etc), as observed in many parts of India. Therefore, an interdisciplinary approach may not prosper if the researchers restrict themselves in their discipline specific attitudes.

In such conditions, community specific social science approaches seem to be more useful to analyse the issue. Social counselling and cultivation of more advanced lifestyle may eradicate such issues at its root. However, with high social science motivated approaches, interdisciplinary approaches may be considered as “soft” and lack in consistency or ideology may be lost to find out a core reason in such social issues. For example, more social science approaches to study the dowry issue may lead to a conclusion from socio-cultural views which lack evidence based assumption that low income of people is the main factor for collecting dowry in marriage. Such dogmas place great barriers in the career paths of workers who offer interdisciplinary approaches to solve problems. Under such conditions, the work gets affected from its grass root level. For example, interdisciplinary proposals applied for grants are often executed by peer reviewers from established discipline specific experts not surprisingly from interdisciplinary researchers. As a result, the applicant experiences trouble in getting funding for their research. Therefore, many time a contractual or untenured researcher on the verge of promotion or regularization of tenure, suspect that evaluators will lack expertise, commitment to interdisciplinary studies. So, a fear factor gives lack of commitment in their mind to carry out interdisciplinary research that may escalate the risk of being denied tenure or restriction in promotion.

At organisation level, interdisciplinary studies may fail if an insufficient self-government system is not offered. Unnecessary directions or interference in their autonomy lead to unsuccessful launch and run of any interdisciplinary program in any organisation and even similar failure may be noticed at professional level. For example, experts or faculties in interdisciplinary programs are usually recruited on the basis of a joint venture, assigning tasks in two or multiply program (such as women's studies (applied and need based program) with history (a traditional discipline), biotechnology and clinical diagnostics (both are need based applied sciences) and philosophy (a social need based predictable discipline) with clinical science (applied health science). However, the last case is little confusable how a social science can be merged with biological science, the central story of this article and is discussed earlier. Post interdisciplinary study barrier includes another boundary for publication of the results. Most of the journals are highly discipline specific and also that too with not a very broad area within the subject. It makes the interdisciplinary researchers very difficult to publish their results. Although journals such as “Measurement: Interdisciplinary Research and Perspectives”, Scientific Report, Social Welfare: Interdisciplinary Approach are many emerging Journals emerged in the last few decades, yet they seem to be insufficient to cover all the results in their area. Establishment of reputed journals covering both the social sciences, pure sciences and most importantly interdisciplinary results covering humanities and science are highly needed in the present day society. It makes the organisation very difficult to compete with the traditional organisations. In addition to the above restrictions, budgetary provision for traditional universities and organisations are always well channelized than the newly established interdisciplinary organisation. This makes it very tough to account for a given scholar or salary of facilities and organisation associated expenditures. Finally it leads to a very restricted boundary to establish interdisciplinary courses in existing and newly established organisations (Clark and Wallace, 2015).

According to Repko (2008) during summer or winter schools also, pupils must be exposed to a diversity of interdisciplinary based subjects, methodologies and tools and techniques with models. Such short term schooling can be used as a model to test various hypotheses on interdisciplinarity. Methods and tools (for example, entropy and probabilistic methods) exclusively interdisciplinary must be explored with network/graph/statistics methods, case based models etc. with live events). And finally engaging students in group or community based programs with interdisciplinary tools outside the familiar domain of experience, such as class room or laboratory may develop their skills to a better extent. Although, no guarantees can be given that such activities will engage pupil's interest in interdisciplinarity or will elevate their understanding of it; the short term of summer school itself can be definitely useful to modulate the studied variables to enhance the efficiency of pupils on interdisciplinarity. And, varieties of experiments on pupils can be done to establish interdisciplinarity in them. As a result, diverse approaches with tactics can be the key ingredient in the course content as per the society and pupils interest, in pedagogy. The evolution of pedagogy thus can be obtained by making interaction with students, communities, societies, and societal issues to schedule a solution based interdisciplinary study. It will develop long lasting curiosity among students in participating interdisciplinary studies, and their positive response will add to their experience for research on societal issues with interdisciplinary approaches. It will definitely make them able to shape their knowledge, skills, involvement with society or community to sharpen their expertise on interdisciplinary. Then they may serve as examples for the future summer school aspirants, and can be used as seeds for spreading the charm of interdisciplinarity for the next generation.

The important steps under this course would be, to define the problem or state of community or society and to focus on the issue based question(s), to justify working on the issue with an interdisciplinary approach, to identify relevant disciplines to merged to address the issue, to conduct a literature search on the problem, to develop competence in each relevant disciplines before the course of action (i.e. research) is started, to analyse the problem and evaluate each insight to it for resolution with interdisciplinarity, to integrate the obtained insights and to produce an interdisciplinary understanding, to identify conflicts between or among thoughts, concepts, perception and their root causes, and finally to discover common statements of the societal issue(s) in terms of interdisciplinary words. Finally to solve the issue by interdisciplinarity with community interaction and outreach program (Repko, 2008). However, a pre-planned course of action or pedagogy is needed to obtain success using summer or winter school as a model.

At cultural level, there are also limitations that restrict the boundary of interdisciplinarity. For example, there is a provision of marriage in blood relation in a Telugu community in both Andhra Pradesh and Telengana states of India. In their community, siblings from brother and sisters are allowed to marry (Paul and Spencer, 2008). Marrying within a family can lead to abnormalities in siblings. It is because, the genes that are not responsible to create any genetic disease when absent or present in a single copy in a person becomes double in the offspring when two blood relation couples get married, each having single copies of the gene. For example, sickle cell anaemia, a deadly genetic disease that occurs in a person when two dominant copies of the gene namely “S” are present in double copies. It means when a person has genetic makeup as “SS”, and the person contracts the disease, however, in a condition where the combination of “Ss” (s being the recessive copy of the gene), “ss”, and the person does not contract the disease. On the other hand, in a condition of “Ss”, the person acts as a carrier of the disease Therefore, when both the persons in a couple are with a genetic makeup of “Ss”, 25% of their children contract the diseases and 50% of them again becomes the carrier of the disease (Griffiths et al., 2012, Figure 4). Therefore, it is strictly advised to not allow marriage between blood relations. All know such scientific blunder but still allow such marriages. And it is their culture which does not allow having an interdisciplinary approach to fix the issue.

**Figure 4:** Social customs and scientific issues. Blood relation marriage and higher risk of transmission of genetic diseases, for example, sickle cell anaemia.

Another example is unusual behaviour of the residents from Swabhimanarea, Malkanagiri, Odisha state, India where they do not consume, even do not know how to use milk and milk products. Although they profusely rear cattle, milking from cows is done in minimal amounts only for the purpose to worship god. Their children undergo severe food security issues including malnutrition but they never feed either milk or milk products to them. Reasons are highly cultural and inherited from their ancients, as opined by few of the residents (Odishatv, 2019). So, a social approach may first explore the solid reason behind such cultural issues, followed by a scientific intervention via audio, video and awareness that can be done to make the residents to consume milk. Their genetic and biochemical analysis may provide the clue how their immunity is mediated without milk meal, could be the new scientific interpolation. Another such cultural issue exists in the Meghalaya state of India, people being resistant to allow railway expansion to their area. The connecting railway project between Tetelia (Assam state) and Byrnihat (Meghalaya state) has remained suspended due to the protest by the residents of Meghalaya. Shillong, commonly called as the "Scotland of the East" and the capital of Meghalaya state has one of the most attractive tourist spot, although tourist and the residents have to travel by only on road to this beautiful hilly town anchoring Cherrapunji, credited being as the wettest place on Earth, aside. The transporting stops in night thereby; it pulls many tourists to trouble (TST, 2019). This is a national social issue in India and the main trajectory to solve the issue to council the “Khasi”, “Garo” and “Jaintia” tribe, being its dominant resident (~35%, 30% and 19% of total population, respectively) that connecting train route into their city would not efflux outsiders to dilute their culture. So, the social insecurity that arrived in their mind from the last few decades needs the intervention of social scientists first followed by legal protection and scientific intervention to modernise them.

Due to the above barriers but not limited to those only, interdisciplinary researchers are highly motivated to become discipline specific. Therefore, the research area from interdisciplinary subject become again discipline specific by keeping their parental subject in dominated condition such as neuroscience (dealing with neural biology), cybernetics (the science of communications and automatic controlling between or alone in machines and living things), biochemistry (explanation of biology in terms of chemical stoichiometry and molecular level), and biomedical engineering (using tools of engineering in clinical and biological sciences). Although terms like economic zoology, seem merging economics and zoology, it deals with more zoology and really nothing about the core concepts of economics. Similarly, clinical sociology needs to be practised with medical practitioners, community health service providers, and social policy and public health campaigns. However, terminology or interdisciplinary subjects such as philozoology (merging philosophy and zoology, possible definition” branch of interdisciplinarity that deals with study of animals from philosophic concepts such as happiness, reason, nature, progress, and liberty), philobotany (merging philosophy and botany, possible definition” branch of interdisciplinarity that deals with study of plants from philosophic concepts such as happiness, reason, nature, progress, and liberty. This branch may strictly deals with plants that really form a good association to grow faster for better production to meet the current day high need of food security), sociozoology (merging sociology with zoology, possible definition: branch of interdisciplinarity that deals with study of animals or especially human from philosophic concepts, biopolitics (merging biology with politics, possible definition: branch of interdisciplinarity that deals with maintaining or conceptualise for the optimal and fine tune in human social race (like euthenics and euphenics: deals with changing conditions to alter the negative impact of a person's genetic problem, means, genetic manipulation for production of a better human race (Baron, 2019), to evolve extraordinary devoted politicians), chemicosociology (merging chemical sciences with sociology, possible definition: branch of interdisciplinarity that deals with study of discovery, social acceptance and subsequent use of biocompatible chemicals, for example, polyanhydrides, hyaluronan, chitosan and hydroxyapatite, that are used as biomaterials (Pandey et al., 2016), and at least but not last the most essential terms “genosociology” or “genophilosophy” (merging the branch of genetic engineering with sociology or philosophy, possible definition: branch of interdisciplinarity that deals with study of discovery, social acceptance and subsequent use of genetically modified crops and animals and their acceptance in society, this is a very complicated issue in many countries such as India where huge social constraints are set by many socialist and non-biologists against the use of genetically modified crops such as BT Brinjal) and use are not being used or least used elsewhere. These emerging disciplines are occasionally considered as "interdisciplines". Conversely, even though current pedagogy in different institutions or organizational and social entities is focusing on interdisciplinarity, complex and unique hurdles, severe criticisms and disapproval are discouraging. So, the obstacles and challenges faced by interdisciplinarity goals can be learnt from the past two decades and need to be resolved at "professional", "organizational", and "cultural" levels (Ali, 2011).

Interdisciplinarity can be developed with differences in depth, borrowing of concepts, methods, problem oriented collaboration that moves across the disciplines as a result a new inter-discipline emerges. Interdisciplinary research processes require extra skills and efforts for bridging the barriers between or among the different disciplines. Methods for supporting the interdisciplinary research process could be conceptual analysis, articulation of assumptions, etc., research process model, dialogue across scientists and humanists and finally to develop toolbox projects (Keestra, 2013). To achieve interdisciplinarity, acquaintance to a variety of disciplinary works, tools, techniques must be the prerequisite. Some of the basic mandate to be interdisciplinary in nature must include proficiency on the language (to use it as mode of communication and transmission of ideas), on ontology (to collect a set of objects on the concepts and categories in a discipline or domain that shows interrelations), on epistemology (to know the composition of the knowledge on the discipline and to gain the skill to acquire and validate the obtained knowledge), on theoretical perspectives (to gain broad idea about the societal issues), on practical concepts (to collect basic information on the issue in community using methods and tools, on data (to be collected and analysed) and finally on valid norms for acceptability to deduce a solution (Jacobs, 1989). The end result must give a value added knowledge based society. Minimum two major steps are required to have successful interdisciplinary research. First, drawing on disciplinary insights and second, integrating insights and producing an interdisciplinary understanding. Meanwhile, designing and testing for implementation of interdisciplinary curriculum is also important to achieve success in interdisciplinarity. The interdisciplinary curriculum must be based on the growth of knowledge, fragmented schedules (of curriculum), society's response to fragmentation, relevance to the present day society, and definitions that clarify practice and most importantly the merging score of humanities with science, not among disciplines from science and or humanities alone (Jacobs, 1989).

Terminology such as cross disciplinary (Turna and Bolat, 2016), interdisciplinary (Piaget, 1972), pluridisciplinary (Piaget, 1972) and transdisciplinary (Turna and Bolat, 2016) are also used in parallel to achieve the common but emerging complex goals of society. Therefore, it is rightly quoted that “Future-proofing undergraduates begin with an interdisciplinary skill set” (Fidoe, 2019). And, may be a higher pace in interdisciplinarity could be the call of the future especially in developing countries such as India.

Owing the call for interdisciplinarity, many approaches are made especially in clinical sciences to use interdisciplinary mode. For example in nursing (Smith et al., 2019), paediatrics (Liossi et al., 2019), dental sciences (Didilescu and Martinez-Sanz, 2019; Guzmán-Armstrong et al., 2019), neural and dementia management (Rodriguez et al., 2020), even in clinical awareness programs including COVID-19 awareness (Sentell et al., 2020), use of interdisciplinary mode is suggested. In educational hubs such as in biochemistry and molecular biology (Macaulay, 2019), social psychology (Sinha, 2019), interdisciplinary framework is highly recommended even for undergraduate students (Tripp and Shortlidge, 2019). Interdisciplinary studies are also suggested that it has tremendous implication in agriculture sectors especially in soil science management (Hou et al., 2020), disaster management (Gilligan, 2019) especially in hurricane related researches (Murray-Tuite et al., 2019). A simulation based research indicates that interdisciplinary education is much better than disciplinary education Bullard et al. (2019). However, educational systems are yet to employ such approaches evenly across the world.

All above discussion concludes that both science and humanities have their own advantages, acting as two sides of a coin for human society and highly essential for resolving various contemporary issues. Humanities are the basic subjects needed to nurture the human life while science gives a reality to human life. The later one is always changeable. It is because the scientific methods are not fixed but all the time they grow and are developed into a need based purposeful process, as has been well described by J.D. Bernal in Science in History in 1968 (Hodgkin, 1980). Such plausible definition and usage principle of science in relation to human life goes to the credit of the French philosopher of science and founding sociologist, Auguste Comte, who wrote the fact about science in the text series “Compte in Cours de philosophie positive” published in between 1830 to 1842 (Bourdeau, 2011). He opined that human behaviour must be involved with the laws of sciences and humanities to have better life (Bourdeau, 2011). Additionally, science as a phenomenon exists independent of human consciousness and is the most objective thing widely known. However, science in the making is as subjectively constituted as any other branch of endeavour in any discipline, as stated beautifully by Einstein in “Maxwell's Influence of the Idea of Physical Reality in 1940” (Einstein, 1931). This is what we observe in Wilhelm Dilthey, a philosopher and historian of culture, wrote six-volume of translation series (1833–1911) “Introduction to the Human Sciences of 1883” (Dilthey, 1989). He had a strong elaborated on the 20^th^ century interdisciplinary move. It is because, the interdisciplinarity addresses the relationship between power and knowledge used for social control measures (Figure 5).

**Figure 5:** Model explaining the association between science and humanities in interdisciplinarity. Multidisciplinary may be set on the basis of contemporary and future societal needs that should lead to flexibility in holistic education and in turn it would develop ethics, constitutional values, creativity, critical thinking, problem solving, philanthropic participation in pupils. Multidisciplinary must primarily address the relationship between power and knowledge, and how they are used as a form of social control through societal institutions and a critical history of modernity for better problem solving of contemporary issues. All these could be better possible with multidisciplinary approaches rather than a disciplinary approach.

**Figure 6:** Self-explanatory figure displaying the need of pace in interdisciplinary work to solve regional, national and international issues.

Probably, owing to the advantages of interdisciplinary education, the Ministry of Human Resource Development, Government of India, New Delhi, has adopted a New Educational Policy (NEP), implemented recently in August first week. The NEP has focused on multidisciplinarity. It indicates that Indian Institutes of Technologies (IITs), the premier category institutes of India imparting quality education and research, will become multidisciplinary institutions (MHRD, India, 2020). The plans will especially open doors for humanities students into IITs, although few of the IITs already have this system. As a result, students from humanities can be trained in science subjects, as IITs offer the choice based credit system to their pupils in a very flexible manner. The engineering based institutions, such as IITs, should move to adopt more holistic and multidisciplinary approaches of education with more disciplines from arts and humanities (MHRD, India, 2020; Nandini, 2020). Also, as a part of amendment in NEP (2020), Indian universities and colleges will follow multidisciplinary mode education that will offer undergraduate and graduate programmes, with high quality teaching, research, and community engagements of students under a single roof. The 4 year multidisciplinary Bachelor's programme, however, was recommended as the preferred option. The plan is also included in NEP to open at least one large multidisciplinary institution in or near every district by 2030. The NEP also offers that by 2040, all higher education institutions of the country shall aim to become multidisciplinary institutions having a capacity of 3,000 or more students (Nandini, 2020).

The end of the story must rely on the fact that humanities are the origin of many disciplines such as language subjects (considered as the first discipline based on which other disciplines heavily rely) act as the base of every discipline and belong to humanities. Without language skill, many disciplines are under presented. Similarly, studying the existing issues in society can be well analysed and confirmed using approaches from social science disciplines. Then the issue(s) may require approaches from science discipline or from both the disciplines to be carefully and fully addressed. Therefore, equal or due credits to each discipline irrespective of their origin must be given. Every discipline must be useful to create a better world and for the betterment of human beings.

## 6 Conclusion

The purpose of science is to know about either physical and natural objects or the world through observation and experiments. The main objective of science is to understand the mechanism underlying any worldly object but strictly not restricted to it, for example, studying objects out of world i.e. space science. So, the real definition of science is nothing but an extension of human need based practices that co-existed from (pre-) historic time to till now. Initial perceptiveness on societal issues reveals that the humanities and science are quite compatible to outline interdisciplinarity. Humanities are the use of approaches which are predominantly hypothetical but critical, and have a noteworthy historical component, and this methodical aspect distinguishes it from the mainly experiential approaches of the (natural) sciences. So, humanities subjects are analytical in nature while science is based on empirical observations. However, the basic approaches in both humanities and science remain the same that both of them need a hypothesis, sound methodology, and interpretation of data for the practical use in society. Therefore, the end user of the interdisciplinary studies is human in both the cases. So, only interdisciplinary research must not be focused on the core subjects of science. For example, philosophy discipline can be a part of science or vice versa can be true. It is concluded that the present day need is highly aimed for interdisciplinarity along with individual subject research to solve the critical issues of the society (Figure 6). Especially, India, as a bright example of developing countries, such interdisciplinary collaborations across the boundary are highly wanted. Both researchers across disciplines such as from both science and humanities and funding agencies must give due importance for the interdisciplinarity on priority basis.

## Declarations

### Author contribution statement

All authors listed have significantly contributed to the development and the writing of this article.

### Funding statement

This work was supported by The Science and Engineering Research Board (ECR/2016/001984), the 10.13039/501100010803Department of Biotechnology, DST, Government of Odisha (1188/ST, Bhubaneswar, dated 01.03.17, ST-(Bio)-02/2017) and the State Odisha State Higher Education Council, Dept of Higher Education, Government of Odisha (OURIIP Scheme, 1076/69/OSHEC, 26.11.19), India.

### Data availability statement

No data was used for the research described in the article.

### Declaration of interests statement

The authors declare no conflict of interest.

### Additional information

No additional information is available for this paper.

## Appendix A Supplementary data

Supplimentary file Supplimentary file
